# Microarray based comparison of two *Escherichia coli *O157:H7 lineages

**DOI:** 10.1186/1471-2180-6-30

**Published:** 2006-03-15

**Authors:** Scot E Dowd, Hiroshi Ishizaki

**Affiliations:** 1 Livestock Issues Research Unit, USDA-ARS, Lubbock, TX, USA; 2 Department of Grazing Animal Production, National Institute of Livestock and Grassland Science, Nasushiobara, Tochigi 329-2793, Japan

## Abstract

**Background:**

Previous research has identified the potential for the existence of two separate lineages of *Escherichia coli *O157:H7. Clinical isolates tended to cluster primarily within one of these two lineages. To determine if there are virulence related genes differentially expressed between the two lineages we chose to utilize microarray technology to perform an initial screening.

**Results:**

Using a 610 gene microarray, designed against the *E. coli *O157 EDL 933 transcriptome, targeting primarily virulence systems, we chose 3 representative Lineage I isolates (LI groups mostly clinical isolates) and 3 representative Lineage II isolates (LII groups mostly bovine isolates). Using standard dye swap experimental designs, statistically different expression (P < 0.05) of 73 genes between the two lineages was revealed. Result highlights indicate that under *in vitro *anaerobic growth conditions, there is up-regulation of *stx2b*, *ure*D, curli (*csg*AFEG), and stress related genes (*hsl*J, *csp*G, *ibp*B, *ibp*A) in Lineage I, which may contribute to enhanced virulence or transmission potential. Lineage II exhibits significant up-regulation of type III secretion apparatus, LPS, and flagella related transcripts.

**Conclusion:**

These results give insight into comparative regulation of virulence genes as well as providing directions for future research. Ultimately, evaluating the expression of key virulence factors among different *E. coli *O157 isolates has inherent value and the interpretation of such expression data will continue to evolve as our understanding of virulence, pathogenesis and transmission improves.

## Background

Kim et al., [1] utilized octamer-based genome scanning to evaluate genome diversity among *E. coli *O157 isolates. Based upon this genetic fingerprinting method they noted two distinct lineages of this pathogen, one of which tended to cluster the majority of human isolates utilized in their study, and the second which grouped together isolates primarily of bovine origin. They suggested that one of these lineages (Lineage II) may not efficiently transmit to humans from bovine sources. Pradel et al. [2] also found that there were distinct lineages among isolates derived from patients with hemolytic-uremic syndrome (HUS) when evaluated genetically using a combination of *stx2*-RFLP (restriction fragment length polymorphism analyses), *stx2 *variant, and plasmid profile analyses. They also suggested that there may be a separate lineage, which was more virulent for humans, along with a lineage, which may not be as pathogenic. Yang et al. [3] utilized a lineage-specific polymorphism assay consisting of 6 genetic markers and found that they could differentiate two lineages of *E. coli *O157 indicating that the occurrence of these two lineages may be widespread. Barkocy-Gallagher [4] using *Xba1 *RFLP analysis also found distinct clusters of *E. coli *O157, including a cluster where most isolates lacked flagella and *stx1 *genes, leading them to suggest the potential for the existence of clustered isolates having differential abilities to cause disease.

The expression of several virulence factors in relation to the existence of two lineages of EHECs have been evaluated as well. McNally et al. [5] found clear differences in the expression of locus of enterocyte effacement (LEE)-encoded factors between different strains. It was found that, *EspD*, when used as an indicator of LEE expression, was expressed at higher concentrations in the majority of strains that were of human origin (15 of 20) compared with only a few (4 of 20) isolates that were of bovine origin (P < 0.001). They concluded that a subset of *E. coli *O157 isolates (*stx*^+ ^*eae*^+^) in cattle were capable of causing severe disease in humans. Another study evaluating gene expression conducted by Richie et al., [6] found that HUS derived isolates expressed higher concentrations of *stx2 *than bovine derived isolates.

Based upon the proposed existence of a less pathogenic lineage of *E. coli *O157, it has been postulated that much of the Class I recall of millions of pounds of meat annually [7] might be greatly reduced. However, even if a separate lineage of *E. coli *O157 (conclusively proven not to cause disease in humans) were identified and concrete methods for differentiating this lineage developed, it would still be unlikely (because of liability issues) to have the suggested impact on the meat industry. Yet, the study of genetic differences between two lineages of this pathogen that possess different virulence or transmission potential could still have wide ranging and significant economic or scientific benefits. For example, if a specific lineage could be more readily eradicated during the farm to fork process, based upon their genetic differences, this might indirectly have the originally intended effect of reducing the volume of Class I recalls. In addition, from a purely scientific standpoint, clues as to why certain isolates may be more pathogenic or more easily transmitted, based upon genetic differences, is of obvious importance in the study of virulence.

## Results and discussion

Microarray analyses, validated by quantitative PCR, showed that, of the 610 genes on the array, 179 genes were consistently and differentially regulated between the two lineages. Of these 179 regulated genes, 73 transcripts showed statistically significant (p < 0.05) differences in expression of greater than 1.2 fold (Table 1 and Table 2) between each member of the two lineages. Table 1 shows those transcripts whose expression was greater (P < 0.05) in each of the LI isolates. Three heat shock and one cold shock protein transcripts were the most upregulated in the LI isolates compared to the LII. In LII isolates cyoE, hscA, and fimbrial subunit 1 were most highly upregulated compared to LI. Table 2 shows those transcripts whose expression was statistically higher (P < 0.05) in each of the LII isolates. Six transcripts that exhibited enough expression difference to be evaluated by CT using quantitative PCR were chosen at random from these 73 and Q-PCR performed as a validation method. These included *ure*D, cyoE, hscA, nrfB [see Additional file 1], chap4, and *stx*2B. Results of Q-PCR were found to agree in each instance with the results of the microarray experiment. Supplementary dataset 1 [see Additional file 1] provides a listing of the 106 genes that were shown to be consistently up-regulated or down-regulated as part of the microarray experiment, but which did not fully meet the stringent selection and statistical requirements additional supplemental dataset 2 provides all the genes on the array.

Results of the microarray experiments showed that the LI isolates express higher transcription of *ureD *(Table 2), as well as *ureA*, *ureB*, *ureC *(supplemental data), compared to LII. In addition stx2B (Table 2) and stx2A (supplemental data) transcripts are detected in higher abundance in Lineage 1. Lineage I also exhibits up-regulation of key fimbria related transcripts, especially *fliC*, *fliT*, and *fliP*. Other attachment related transcripts *csgA*, *csgF*, *csgE*, and *csgG *(curli) were also up-regulated, which could also be highly significant in promotion of pathogenesis [8-12]. When using all of the regulated genes as a single data set for Gene Ontology [13] based analyses, it was found that, up-regulation of genes associated with regulation of urease activity, GTP binding, metabolism, nitrogen metabolism and regulation of transcription were statistically (p < 0.05) more represented in LI isolates (Table 3). In LII isolates peptidase activity, transferase activity, and DNA binding activity were statistically more represented (p < 0.05). These differences could point to a fundamental difference in the environmental response and control networks of these lineages that promotes survival and differential expression of virulence attributes in response to specific environments and hosts. These types of control networks could be the key to understanding differential virulence or transmission potential if such a phenomenon could be proven to exist within the O157 serogroup.

### Stx2

The role of *stx2 *in pathogenesis is well accepted [14-18] and up-regulation of constitutive stx2 expression in the hypothesized more pathogenic LI isolates may not be a surprising finding. The up-regulation of *stx2B *and *stx2A *[see Additional file 1] transcripts is accompanied by up-regulation of regulatory genes associated with Stx2 expression. A complicated network of interactions between the o*raA *(r*ecX*), *dinI*, *lexA*, *umuD*, SSB, *recA*, *psiB *and possibly other unidentified proteins, act in the regulation of RecA function. The role of *recA *as part of an SOS response is to cleave repressors that in addition to the SOS response ultimately lead to Stx2 production [19]. *OraA *(also known as *recX*) and *dinl *are coregulators (competing regulators) of *recA *[20] and both were up-regulated in LI isolates along with the *stx2 *subunit transcripts. *OraA *is thought to be co-transcribed with *recA *during SOS response [21]. *RecA *specific oligos were not included in the array but we might expect that being co-transcribed along with *oraA *that it would likely be up-regulated in LI as well. *PsiB*, (supplemental) is also up-regulated in LI and thought to prevent ssDNA from inducing an SOS response by inhibiting activation of *recA *protein [22]. *PsiB*, is found on many conjugative plasmids near the origin of conjugative transfer and has anti-recombinase activities [23]. Expression of the *dinI *protein of *E. coli *inhibits both the co-protease and recombinase activities of *recA *in vivo [24]. Yet, in spite of all of the regulators of SOS response in LI isolates, we still observe a significant up-regulation of *stx2a *and *stx2b *transcripts which have been shown to be expressed as part of an SOS response [25-27].

With up-regulation of *dinl*, *psiB*, *oraA *and also with the up-regulation of *stx2a *and *stx2b *and various other genes related to stress response it could be an indication that LI isolates do have differentially regulated pathways the enhance its toxin expression potential. It does appear that the current LI isolates have a modified regulatory system response, which significantly promotes Stx*2 *toxin production compared to LII isolates. We have also considered that LII isolates may have mutations affecting the integrity of the *stx2 *prophage's late regulatory transcripts shown to encode *stx2 *[28-31]. Future work looking at the actual Stx*2 *toxin levels as well as evaluation of the structural integrity of the Stx2 phage in these 6 isolates via sequencing or PCR would be a beneficial follow up to this research. We have performed Stx2b specific ELISA and quantitative PCR analysis of 20 additional LI and 20 additional LII isolates as part of a follow-up study, and found that the LI isolates have statistically (p < 0.05) higher transcription rates and protein concentrations under these same conditions (data not shown). If these LII isolates have a defective toxin production system this could be a strong indication that they lack one of the key virulence factors contributing to the pathogenicity of O157 [15,16,32-34].

### Urease

Enterohemorrhagic *E. coli *has been shown to be highly adaptable to various extreme environments (water, heat, freezing, acid, desiccation, hypo- and hyperosmotic, disinfectants etc) which contributes greatly to its success as a pathogen [35-46]. To succeed as a enteric pathogen with a low infectious dose [47-49], *E. coli *O157 must be able to survive passage through the acidic environment of the stomach if they are to cause gastrointestinal disease [50]. As an indication of their evolutionary focused ability for surviving acidic environments they possess 3 acid resistance pathways [51] and urease could act as an additional system to modify anion concentrations. Therefore the up-regulation of urease in LI isolates is of interest in spite of recent work indicating that *E. coli *O157 has only rarely been shown to exhibit urease activity [52-55]. As an example, a previous study noted that lack of urease activity in EHEC strains is often due to a base substitution in the *ureD *gene causing an early termination of the transcript [54]. Urease expression and activity be condition, host, or environment specific and could be expressed only in specific environments to beneficially modify internal and/or surrounding anion concentrations, enabling EHEC to survive acidic conditions and contributing to its low infectious dose. Thus, environmental (bovine) isolates may not possess or have sufficient selective pressure for maintenance of detectable levels of urease transcript expression under the conditions evaluated.

Previous research by Heimer et al [52] suggests regulation of the urease operon is through *fur *(not differentially regulated) and an unknown trans-acting factor. It was hypothesized that this transacting factor is missing in *E. coli *O157:H7 strain EDL933 (atcc # 43895) though other O157 strains (IN1 and MO28) have been shown to possess some urease activity. However, none of the isolates showed differential regulation of *fur *which may be an indication that the LI isolates may be differentially expressing this proposed transacting factor, which is promoting up-regulation of the urease operons under the current growth conditions. It is likely that based upon previous evaluation that there is some low level urease activity that is not evident in *E. coli *O157 strains using conventional methods such as Christensen agar [56]. We have begun investigations of the effects of pH, different laboratory media, anoxia, nickel supplementation, and cytosolic specific urease based acid resistance assays on the ability to detect urease activity in O157 isolates.

### Curli

Several factors related to attachment are up-regulated in LI isolates. These include curli fibers, type III secretion apparatus genes. This suggests that LI isolates have constitutive up-regulation of many genes that are involved in intimate attachment. It was reported that curli fibers are infrequently expressed during in vitro growth of *E. coli *O157:H7 [8] and that strains containing variations at the *csgD *promoter region, which induced expression of curli, are associated with increased virulence in mice and increased invasion of HEp-2 cells [57]. In this experiment there was significant up-regulation of *csgA *and *csgD *as well as some evidence for up-regulation of the both *csg *operons [see Additional file 1] in the LI isolates compared to LII, yet genes involved in regulation of curli operons do not correspond to this observation. *RpoS *has been shown to interact with *hns *(neither differentially regulated) to derepress *csgAB *expression [58]. Further contradicting the increased expression of curli operons in LI, *ompR *is up-regulated in LII. Increased *ompR *expression has also been associated with increased curli production yet a single point mutation, in *ompR *[59]. Future work should likely evaluate whether curli fibres are actually being produced and assembled under these *in vitro *conditions in LI isolates.

### Virulence gene regulation

One of the more interesting of the up-regulated genes in LI is *rfaH*. Originally, discovered as a primary regulator of LPS-core synthesis in *Salmonella enterica *and *E. coli *[60,61], *RfaH *is noted as a primary virulence regulator of *E coli *that functions as a transcriptional anti-terminator [62,63] in long operons. These operons include those encoding the F-factor, O-antigens, different capsules, hemin uptake receptor, alpha-hemolysin, and CNF-1 [64-73]. Inactivation of *rfaH *in uropathogenic *E. coli *has be shown to inhibit pathogenicity completely [74]. *RfaH *mutants have been shown to have reduced ability to survive/grow in the presence of bile salts [75]. The up-regulation of *rfaH *in LI isolates may be an important avenue to pursue as a means to explain their hypothesized enhanced virulence.

### LEE

LII isolates showed an increased expression of *toxB *which is known to promote expression of genes encoded by locus of enterocyte effacement (LEE). Indeed, several of the *esp *(*A, B, P*) showed slight cumulative up-regulation. In addition, most of the *etp *genes involved in the type II transport system were also up-regulated. The type II secretion system was recently noted as also being involved in intimate attachment through secretion of *stcE *[76]. These results showing upregulation of such an important virulence factor in LII isolates points out two key features that are of importance in this manuscript. The first is that these results as intended can help with identification of isolates which may serve as good regulatory models for providing additional insight into virulence expression. In addition, these results are obviously counter to the overall hypothesis that LI is either more virulent or has more potential for transmission and therefore serve as a caution for the interpretation of results. Thus, as with all microarray studies care must be taken in interpretation of the results, yet negative results or results counter to the hypothesis should not be ignored.

### LPS, fimbria, and Flagella

LII isolates also show notable up-regulation of genes involved in a number of systems that are noted as virulence factors. Of interest in LII is the comparative up-regulation of LPS, fimbria (FimH), capsule, and flagella related genes (Table 1 and supplement). Considering that the isolates were grown under anaerobic conditions the increase in LPS and flagella related transcripts represents what may be a typical K-12 like *E. coli *response to anoxic conditions [77] in the LII isolates, while the LI seem to be lacking this common profile. The hypothesized decrease virulence of LII may be partially explained by the more pronounced regulation of certain virulence factors by LI. Another interesting aspect that is related to the expression of genes associated with motility and the results seen here is the hypothesis proposed by Monday et al. [78], which is related to a competitive interaction between different type III secretion systems. According to this hypothesis there could be a competitive interaction between the type III secretion systems associated with flagellar export and assembly and the type III secretion system that mediates the injection of virulence factors (LEE). Thus, because O157 has multiple type III systems there is the potential for these systems to interfere with one another. This competition could ultimately affect the expression of motility and/or virulence factors. Thus, because there is an increase in LEE expression as well as motility genes in LII isolates it may be a result of an interaction of the type III regulatory networks in these isolates.

In proper proportions type 1 fimbriae and the LPS of uropathogenic *E. coli *are known to operate together to induce apoptosis in human neutrophils [79]. The cooperative effects of these virulence attributes may function as a mechanism by which *E. coli *induces infections of the urinary tract. However, if LPS is over produced, excess LPS is likely to be secreted by bacteria into their environment, which may have the opposite effect. In fact, it has been documented that if significant amounts of LPS is released from non-adherent bacteria this has an anti-apoptotic effect on neutrophils, suggesting that LPS can also serve as an important regulator of neutrophil survival in tissue [79]. Up regulation of LPS by LII isolates compared to LI isolates, if this excess LPS were shed from the bacteria, maintained in the cytoplasm, or deposited in excess onto the membrane might also be toxic to the bacteria inhibiting its own growth and interaction with its environment [80]. Overproduction of LPS could also alter bacterial cell morphology by accumulation in the bacterial cytosol, which could also potentially prevent pathogenesis. Previous work [81] and [82] demonstrated that *E. coli *O157 exhibiting reduced production of O157 LPS side chains displayed an increased binding to tissue culture cells. It was concluded that the presence of the O157 polysaccharide has the potential to interfere with the adherence and its expression is not required to produce the attaching and effacing lesions. Excess LPS may act to mask adhesive structures present on the bacterial surface. It is also possible that the physicochemical properties of the cell such as surface charge or hydrophobicity may be altered by lack of or excess LPS. These hypothetical interactions and the effects of LPS expression on pathogenesis are again a highly interesting topic for future research.

## Conclusion

It has been hypothesized by various researchers that a less pathogenic lineage of *E. coli *O157 exists. Geared toward finding evidence that might direct research toward genetic mechanisms that support the hypothesis of differential virulence or transmission potential we evaluated representatives from these two lineages in a preliminary study. The results highlight several of the more important virulence factors as being differentially regulated, as well as various regulatory networks that may provide useful insight and targets for future research. Key virulence factors were shown to be upregulated in LI, especially those that have been suggested to promote virulence and transmission potential. However, other contradictory findings were also uncovered in which several virulence factors more associated with colonization and pathogenesis were also upregulated in LII isolates. Many previous studies describing regulatory mechanisms are supported by the results of this study, providing some additional insight into the control of virulence genes. Though the hypotheses considered as part of this research is still far from conclusive, the results do provide a valuable foundation that will direct future research. Ultimately, evaluating the expression of key virulence factors among different *E. coli *O157 isolates is valuable beyond the reasoning discussed within the confines of this report, and the interpretation of such expression data will continue as the understanding of virulence, pathogenesis and transmission evolves.

All cells have stress response pathways that help to maintain homeostasis, however it appears that these two lineages of O157 may have diverged just enough that their regulatory pathways are geared for different purposes, ultimately promoting survival in different environments and hosts. It is not clear yet, though research is ongoing, whether LII isolates have lower transmission potential or lower virulence or indeed whether there is enough divergence between the two lineages to consider them as separate. One hypothesis presented in the literature and also supported by the data presented is that LII strains may be more co-evolved as a symbiont of cattle, which promotes its long-term survival in this specific reservoir. For instance, stx2 expression may not be as beneficial in colonization of a bovine host as it has been noted that intestinal receptors for Shiga toxin are found in humans but not cattle [83], while LEE island expression may be very important [84]. Popular theories of pathogen evolution suggest that as a pathogen evolves within finite populations, the pathogen tends to become less virulent (attenuation) to the host thereby promoting though various mechanisms of evolution its own transmission and survival among the populations [85]. This may be exemplified by the differential expression of stress response genes, which could prime or maintain an isolate of *E. coli *O157 in a genetic state that is able to rapidly respond to conditions the isolate might encounter during transmission from animal to human hosts, through the farm to fork process, thereby increasing its transmission potential.

## Methods

### Bacterial isolates and growth conditions

A working set of lineage (20 LI and 20 LII) isolates as described in Kim et al. [1] were obtained from A. Benson (University of Nebraska, Dept. Of Food Science and Technology, Lincoln, Neb.). LI isolates 43895, fda518, frik533 and LII isolates ne037, frik2000, frik1985 were chosen at random and utilized in the current analyses. Isolates were grown on LB agar under anaerobic conditions for 12 hours. Previous growth studies noted that these 6 isolates displayed similar growth curves, OD600, and concentration (data not shown). Stationary phase was selected to ensure that all isolates and cultures were at the same stage of growth. Isolates were of the Stx2vha genotype and all exhibited typical O157 phenotype characteristics including acid tolerance, lack of sorbitol fermentation, lack of glucuronidase activity and beta hemolysis on tryptose blood agar (Difco, Sparks, MD) with washed, defibrinated sheep blood (Oxoid, Lenexa, KS). All isolates also displayed the same phenotypes using API20 (bioMerieux, Durham, NC).

### Microarray design

Using the transcriptome of *E. coli *O157:H7 EDL933 an oligonucleotide microarray (~50mer) was designed. Based upon funding available we were able to choose 610 genes [see Additional file 2] including 10 negative control genes derived from pig sequences, which were selected based upon their being associated with virulence or with regulation of virulence genes. Specifications of oligos were based upon various design characteristics such as temperature of melting, 3' location, specificity, lack of repeat nucleotides, etc. [86]. Oligos were synthesized and normalized in concentration by Integrated DNA Technologies Inc. (Coralville, IA). Oligos were resuspended in Epoxide Slide Spotting Solution and printed onto Epoxide Coated Slides (Corning Inc., Corning, NY). Each array consisted of duplicate elements and each slide contained a duplicate array.

### Microarray protocol

All procedures were performed according to respective manufacturer protocols. Colonies were resuspended immediately in RNAprotect Bacteria Reagent (Qiagen Inc., Valencia, CA) after they were harvested. Total RNA was extracted using RNeasy Protect Bacteria Mini Kit (Qiagen Inc.) and DNA removed using RNase-Free DNase Set (Qiagen Inc.). RNA was quantified using a nanodrop ND-1000 device (NanoDrop Technologies, Wilmington, DE) and quality confirmed by electrophoresis. RNA was labeled with either CyDye3-dCTP or CyDye5-dCTP (Amersham Biosciences) using the LabelStar kit (Qiagen Inc.) and Random nonamers (Sigma-Aldrich Inc., St. Louis, MO). Labeled cDNA was hybridized to the microarray using Universal Hybridization Solution (Corning Inc.).

### Microarray analysis

Each microarray experiment was performed in duplicate and each experiment also had a corresponding dye swap for an added technical replication. As an example of a dye swap design LI is labeled with cy3 and LII is labeled with cy5 in one array and in the second array LI is labeled with cy5 and LII labeled with cy3. Dye swaps are not biological replicates but provide technical replication that accounts for different dye incorporation rates. Images were captured using a Genepix 4000B (Molecular Devices Corporation, Union City, CA) laser scanner and images processed using GenePix 6.0 software (Molecular Devices Corporation). Analysis was performed using Acuity 4.0 software as well as GeneSpring 11.0 software (Agilent Technologies, Palo Alto, CA). Results were compared between the two software packages to assure conformity of results. Slides were normalized using standard settings (ratio based so that the mean of the ratio of means, of all features, were equal to 1.0). All ratios less than 0.1 and greater than 10.0 were excluded, as well as bad, low signal, absent, or unfound features. To obtain our final data provided in Table 1 and Table 2 we required that all arrays, duplicate elements on each array, and these same features on the dye-swap experiments (after mathematical conversion x' = -x) to provide agreement, show significant relevance at the p < 0.05 level, and exhibit at least 1.2 fold regulation. A supplemental dataset was derived for those genes that showed a tendency to be differentially expressed. Usually, the lack of inclusion into the stringent dataset was only based upon the quality of the signal in one of the array or dye swap comparisons. Therefore, these results are provided for information and discussion purposes.

### Quantitative PCR

The results of the array were validated using quantitative PCR. Subsets of the regulated genes were chosen at random and primers designed using Primer Select 2.0 software (Applied Biosystems, Foster City, CA). RNA was quantified using NanoDrop system and then using QuantiTect SYBR Green RT-PCR kit (Qiagen Inc.) relative CT was determined with 16s as a control gene, using ABI 7500 Real Time-PCR system (Applied Biosystems).

### Functional analysis

HT-GO-FAT software was used to perform the functional GO related analysis. Functional classifications were determined for the regulated genes using HT-GO-FAT and the LIRU8 database. Statistics for higher represented classifications were also determined using HT-GO-FAT. A dedicated Amigo database was also prepared based upon the microarray and the EDL933 transcriptome and can be found at the above URL.

### Statistical analysis

Acuity 4.0 built in statistics algorithms were utilized for all statistics related to microarrays. One sample t test was used to determine the significantly regulated genes. Random samples assigned by computer generation. Standard methods were utilized for evaluation of quantitative PCR based upon target gene Ct values (number of cycles of PCR before a threshold of detection is crossed) normalized with the Ct value of an appropriate housekeeping gene (fadD) to compensate for variation in initial RNA and cDNA concentrations. The first normalization procedure provides the initial ΔCt value. The sample ΔCt values were then normalized against the smallest ΔCt value identified in the complete data set, termed ΔΔCt. Finally, the ΔΔCt value for each sample was transformed by the function 2^ΔΔCT ^to produce the final gene expression value for each sample. This method allowed for direct comparison of relative gene expression values between isolates. Gene Ontology related statistics were calculated as described by Al-Shahrour et al [87].

## Authors' contributions

SD designed the microarray, conceived of the project and wrote the manuscript, HI performed the laboratory experiments.

## USDA disclaimer

The use of trade, firm, or corporation names in this publication is for the information and convenience of the reader. Such use does not constitute an official endorsement or approval by the United States Department of Agriculture

## Supplementary Material

Additional File 1 Regulated Genes p < 0.2 and > 0.05, This file and dataset contains 105 genes that failed a criteria for inclusion in the primary dataset and their significance test was not less the p = 0.05. Click here for file

Additional File 2 All genes contained in the Escherichia coli O157:H7 virulence array, This file provides a list of all of the genes contained in the 610 gene virulence gene O157:H7 array. Click here for file

## Figures and Tables

**Table 1:** This table presents the genes that were consistently and statistically up regulated in the hypothetically more pathogenic lineage I strains.

**Name**	**average mean log ratio (635/532)**	**average fold increase**	**One Sample t-Test (p)**	**definition**	**accession**
*hslJ*	-2.04	4.10	0.017036	heat shock protein hslJ	NP_287767.1
*cspG*	-1.97	3.91	0.018217	homolog of Salmonella cold shock protein	NP_286926.1
*ibpB*	-1.82	3.54	0.037563	heat shock protein	NP_290325.1
*ibpA*	-1.59	3.02	0.031977	heat shock protein	NP_290324.1
Fimb 10	-1.58	2.98	0.011803	putative fimbrial protein	NP_290361.1
*trxC*	-1.39	2.63	0.018467	putative thioredoxin-like protein	NP_289141.1
*feoB*	-1.31	2.47	0.004959	ferrous iron transport protein B	NP_289949.1
*ureD*	-1.28	2.43	0.038695	putative urease accessory protein D	NP_287085.1
*chap3*	-1.26	2.39	0.030462	possible chaperone	NP_288034.1
*ydeA*	-1.23	2.35	0.026584	putative resistance/regulatory protein	NP_287624.1
*ureD_2*	-1.23	2.34	0.050155	putative urease accessory protein D	NP_287085.1
secret3	-1.09	2.13	0.024694	putative secreted protein	NP_288394.1
*fliC*	-1.06	2.08	0.018058	flagellar biosynthesis; flagellin, filament structural protein	NP_288384.1
*stx2A*	-1.00	2.01	0.021712	shiga-like toxin II A subunit encoded by bacteriophage BP-933W	NP_286976.1
*terW*	-0.95	1.93	0.044205	unknown associated with putative tellurite resistance	NP_286699.1
*rfaH*	-0.93	1.90	0.007198	transcriptional activator affecting biosynthesis of lipopolysaccharide core, F pilin, and haemolysin	NP_290472.1
*phoB*	-0.87	1.82	0.006296	positive response regulator for pho regulon, sensor is PhoR (or CreC)	NP_286137.1
*ureA_2*	-0.81	1.75	0.050244	putative urease structural subunit A (gamma)	NP_287086.1
*helicase1*	-0.71	1.64	0.01929	putative ATP-dependent helicase	NP_288767.1
*yegW*	-0.71	1.63	0.015902	putative transcriptional regulator	NP_288603.1
*ureB_2*	-0.70	1.62	0.038644	putative urease structural subunit B (beta)	NP_287087.1
*typeIIIap7*	-0.66	1.58	0.033765	type III secretion apparatus protein	NP_289424.1
*ycjZ*	-0.61	1.53	0.038253	putative transcriptional regulator LYSR-type	NP_287857.1
*ykgA*	-0.60	1.51	0.000965	putative AraC-like transcriptional regulator	NP_286025.1
*sbmA*	-0.59	1.50	0.050279	sensitivity to microcin B17, possibly envelop protein	NP_286115.1
*YjhS*	-0.57	1.49	0.03404	orf, hypothetical protein	NP_290925.1
*ybbK*	-0.53	1.45	0.037791	putative protease	NP_286238.1
virulense3	-0.50	1.42	0.038974	putative virulence gene	NP_290837.1
*pldA*	-0.49	1.41	0.031981	outer membrane phospholipase A	NP_290453.1
*yejH*	-0.48	1.40	0.008115	putative ATP-dependent helicase	NP_288767.1
*transreg*	-0.34	1.27	0.033811	putative membrane spanning transport protein	NP_286232.1
*hydH*	-0.27	1.21	0.00039	sensor kinase for HydG, hydrogenase 3 activity	NP_290635.1

**Table 2:** This table presents genes that were consistently and statistically up regulated in the hypothetically less pathogenic lineage II strains

**Name**	**average mean log ratio (635/532)**	**average fold increase**	**One Sample t-Test (p)**	**definition**	**accession**
*inaA*	0.57	1.49	0.028507	pH-inducible protein involved in stress response	NP_288811.1
*nupG*	0.60	1.51	0.002513	transport of nucleosides, permease protein	NP_289536.1
*ompR*	0.61	1.53	0.019932	response regulator (sensor, EnvZ) affecting transcription of ompC and ompF: outer membrane protein synthesis	NP_289945.1
*flgC*	0.62	1.54	0.008244	flagellar biosynthesis, cell-proximal portion of basal-body rod	NP_287208.1
*secD*	0.64	1.55	0.050195	protein secretion; membrane protein, part of the channel	NP_286147.1
*recB*	0.75	1.68	0.050257	DNA helicase, ATP-dependent dsDNA/ssDNA exonuclease V subunit, ssDNA endonuclease	NP_289372.1
*hemY*	0.78	1.72	0.045026	a late step of protoheme IX synthesis	NP_290430.1
*fhuA*	0.79	1.73	0.015243	outer membrane protein receptor for ferrichrome, colicin M, and phages T1, T5, and phi80	NP_285846.1
*cheB*	0.81	1.75	0.014779	response regulator for chemotaxis (cheA sensor); protein methylesterase	NP_288320.1
*cutC*	0.83	1.77	0.017209	Copper homeostasis protein	NP_288311.1
*secF*	0.96	1.94	0.033545	protein secretion, membrane protein	NP_286148.1
*wecF*	0.97	1.95	0.021373	TDP-Fuc4NAc:lipidII transferase; synthesis of enterobacterial common antigen (ECA)	NP_290425.1
*frdD*	0.97	1.95	0.042158	fumarate reductase, anaerobic, membrane anchor polypeptide	NP_290786.1
*espP*	1.07	2.10	0.023407	EspP	NP_052685.1
*kfras*	1.08	2.11	0.040371	KfraS	NP_052633.1
*etpJ*	1.10	2.15	0.016101	EptJ	NP_052615.1
*toxB*	1.11	2.15	0.020589	toxin B	NP_052665.1
*fliY*	1.11	2.16	0.001708	putative periplasmic binding transport protein	NP_288381.1
*wzx*	1.22	2.33	0.014144	O antigen flippase Wzx	NP_288543.1
*etpH*	1.28	2.42	0.009559	EtpH	NP_052613.1
*etpO*	1.28	2.43	0.021162	EptO	NP_052620.1
*fumC*	1.31	2.48	0.01514	a late step of protoheme IX synthesis	NP_290430.1
*ydeW*	1.34	2.53	0.001173	putative transcriptional regulator, sorC family	NP_287642.1
*etpI*	1.39	2.62	0.005332	EtpI	NP_052614.1
*etpM*	1.57	2.98	0.000193	EtpM	NP_052618.1
*cspD*	1.59	3.01	0.051261	cold shock protein	NP_286652.1
*oppC*	1.60	3.03	0.009279	homolog of Salmonella oligopeptide transport permease protein	NP_287488.1
usher2	1.66	3.15	0.02289	putative fimbrial usher protein	NP_287650.1
*cspC*	1.67	3.19	0.048484	cold shock protein	NP_288259.1
*etpN*	1.68	3.20	0.015507	EptN	NP_052619.1
*etpK*	1.70	3.25	0.000151	EtpK	NP_052616.1
*rpoB*	1.74	3.34	0.005075	RNA polymerase, beta prime subunit	NP_290619.1
*argT*	1.81	3.51	0.007679	lysine-, arginine-, ornithine-binding periplasmic protein	NP_288884.1
fimberal4	1.84	3.58	0.0179	putative fimbrial protein	NP_290128.1
chaper2	1.86	3.64	0.002084	putative fimbrial chaperone	NP_287649.1
*fumA*	1.88	3.68	0.005453	fumarase C= fumarate hydratase Class II; isozyme	NP_288046.1
*etpL*	1.97	3.92	0.009254	EtpL	NP_052617.1
*rpoC*	2.01	4.04	0.021043	RNA polymerase, beta prime subunit	NP_290619.1
*cyoE*	2.11	4.31	0.027937	protoheme IX farnesyltransferase (haeme O biosynthesis)	NP_286170.1
*hscA*	2.32	4.99	0.012973	heat shock protein, chaperone, member of Hsp70 protein family	NP_289083.1
fimbsub1	2.53	5.79	0.029658	putative major fimbrial subunit	NP_287648.1

**Table 3:** Gene Ontology Biological Processes and Molecular Functions representations for level 4 and level 6, presenting genes from the above tables and supplemental data table grouped into those gene ontology categories shown to be statistically over represented.

**Gene Ontology Classification**	% of total upregulated genes in LI	% of total upregulated genes in LII	p-value
**MOLECULAR FUNCTION LEVEL 4**			
Peptidase activity	0	16.33	0.0059
Transferase activity, phosphorus transfer	6.67	22.45	0.043
DNA binding	42.22	22.45	0.048
**MOLECULAR FUNCTION LEVEL 6**			
Urease activity	12.5	0	0.05
GTP binding	12.5	0	0.05
BIOLOGICAL PROCESS LEVEL 4			
**Regulation of cellular physiological processes**	24.62	8	0.009
Regulation of metabolism	24.62	8	0.009
Nitrogen compound metabolism	6.15	0	0.04
BIOLOGICAL PROCESS LEVEL 6			
**Regulation of nucleobase, nucleoside binding**	30.61	11.32	0.02
Regulation of transcription	30.6	15.1	0.026

the file format, the title of the data, and a short description of the data
